# Untreated Human Infections by *Trypanosoma brucei gambiense* Are Not 100% Fatal

**DOI:** 10.1371/journal.pntd.0001691

**Published:** 2012-06-12

**Authors:** Vincent Jamonneau, Hamidou Ilboudo, Jacques Kaboré, Dramane Kaba, Mathurin Koffi, Philippe Solano, André Garcia, David Courtin, Claude Laveissière, Kouakou Lingue, Philippe Büscher, Bruno Bucheton

**Affiliations:** 1 Institut de Recherche pour le Développement, Unité Mixte de Recherche IRD-CIRAD 177, Campus International de Baillarguet, Montpellier, France; 2 Centre International de Recherche-Développement sur l'Elevage en zones Subhumides (CIRDES), Unité de Recherches sur les Bases Biologiques de la Lutte Intégrée, Bobo-Dioulasso, Burkina Faso; 3 Institut Pierre Richet, Unité de Recherche «Trypanosomoses», Abidjan, Côte d'Ivoire; 4 Université d'Abobo-Adjamé, URES de Daloa, Laboratoire de Génétique Moléculaire et Evolution des Maladies Infectieuses Tropicales, Daloa, Côte d'Ivoire; 5 Institut de Recherche pour le Développement, Unité de Recherche 010, Faculté de Pharmacie, Paris, France; 6 Programme National d'Elimination de la Trypanosomose Humaine Africaine, Abidjan, Côte d'Ivoire; 7 Institute of Tropical Medicine, Department of Biomedical Sciences, Antwerp, Belgium; Foundation for Innovative New Diagnostics (FIND), Switzerland

## Abstract

The final outcome of infection by *Trypanosoma brucei gambiense*, the main agent of sleeping sickness, has always been considered as invariably fatal. While scarce and old reports have mentioned cases of self-cure in untreated patients, these studies suffered from the lack of accurate diagnostic tools available at that time. Here, using the most specific and sensitive tools available to date, we report on a long-term follow-up (15 years) of a cohort of 50 human African trypanosomiasis (HAT) patients from the Ivory Coast among whom 11 refused treatment after their initial diagnosis. In 10 out of 11 subjects who continued to refuse treatment despite repeated visits, parasite clearance was observed using both microscopy and polymerase chain reaction (PCR). Most of these subjects (7/10) also displayed decreasing serological responses, becoming progressively negative to trypanosome variable antigens (LiTat 1.3, 1.5 and 1.6). Hence, in addition to the “classic” lethal outcome of HAT, we show that alternative natural progressions of HAT may occur: progression to an apparently aparasitaemic and asymptomatic infection associated with strong long-lasting serological responses and progression to an apparently spontaneous resolution of infection (with negative results in parasitological tests and PCR) associated with a progressive drop in antibody titres as observed in treated cases. While this study does not precisely estimate the frequency of the alternative courses for this infection, it is noteworthy that in the field national control programs encounter a significant proportion of subjects displaying positive serologic test results but negative results in parasitological testing. These findings demonstrate that a number of these subjects display such infection courses. From our point of view, recognising that trypanotolerance exists in humans, as is now widely accepted for animals, is a major step forward for future research in the field of HAT.

## Author Summary

The existence of a diversity of infection outcomes – ranging from self-cure to asymptomatic, severe or fatal cases – is now widely recognised for most parasitic and infectious diseases. The dogma concerning sleeping sickness, however, is still that infection is 100% fatal. Here we describe a 15-year follow-up of patients diagnosed with human African trypanosomiasis (HAT) in the Ivory Coast but who refused treatment. Our results, based on clinical, serological, molecular, and parasitological investigations, combining diagnostic tools for the field and highly specific and sensitive laboratory tests, constitute the most comprehensive study on the natural evolution of *Trypanosoma brucei gambiense* infection in its human host. At least two alternative natural progressions of HAT to the “classic” fatal disease were identified: a progression to an apparently aparasitaemic and asymptomatic infection and a progression to an apparently spontaneous resolution of infection. We believe that recognising that trypanotolerance exists in humans is a major step forward for future research aimed at identifying human-specific defence and immune mechanisms involved in the control of *T.b. gambiense* infection and thus new candidate therapeutic or prophylactic targets.

## Introduction

Human African trypanosomiasis (HAT) or sleeping sickness is caused by infection of two trypanosome sub-species transmitted by tsetse flies, *Trypanosoma brucei* (*T.b.*) *gambiense* and *T.b. rhodesiense*, with *T.b. gambiense* causing more than 95% of all cases [1]. The disease evolves from an early haemolymphatic phase (first stage, P1) to a meningoencephalitic phase (second stage, P2) when the parasites invade the central nervous system leading to neurological disorders [2]. Whereas some *T.b. gambiense* patients develop a chronic disease (i.e. remaining in stage 1 for several years), others progress more rapidly to stage 2 within several months [3]. In the absence of treatment, HAT is widely assumed to be 100% fatal. Indeed, HAT probably killed more than one million people over the three major epidemics that ravaged the African continent during the twentieth century [2], [4].

Little is known about *T.b. gambiense* infection outcome in the absence of treatment, because usually HAT patients are systematically treated as soon as possible after diagnosis, even in the absence of clinical symptoms, since the disease is potentially fatal and tsetse flies can be infected by feeding on these patients [5]. Although reports on asymptomatic carriers and spontaneous cure have been published, questions on the existence of human trypanotolerance still remain [6], [7], [8], [9]. Among the few recently published studies is the example of 53 HAT patients diagnosed in the Sinfra focus (western central part of the Ivory Coast) in 1995–1996 but refusing treatment. These patients were re-examined several times between 1997 and 1999 in order to convince them to accept treatment [10]. Twenty-nine patients accepted treatment, mainly because of the progressive appearance of neurological disorders. Two patients still refused treatment despite the onset of neurological signs and eventually died. Such courses can be considered as the “classic” fatal progression of HAT. In 1999, among 15 patients who remained untreated, six were still parasitologically positive with only one showing neurological signs. Interestingly, in nine patients, an apparent parasitological clearance was observed, among whom six still had positive results on the card agglutination test for trypanosomiasis (CATT) [11] and three had negative CATT results. Of these patients refusing treatment, three of the six patients who were still parasitologically positive and three of the six still CATT-positive but parasitologically negative in 1999 were re-examined in 2002. All were parasite-negative by microscopy, but PCR-positive [12], suggesting that these individuals carried latent infections.

During surveillance activities in 2004 and 2009, the above-mentioned untreated patients as well as treated HAT patients from the same Sinfra focus who were diagnosed within the same period (1995–1996) were re-visited to assess their parasitological and serological status. In addition, we included other HAT cases diagnosed between 2000 and 2007 in the nearby Bonon focus [13], [14], as we had learnt from the local health authorities that they had not yet been treated. We report here on the data obtained throughout this long-term follow-up period.

Our results, based on clinical, serological, molecular, and parasitological investigations, combining field diagnostic tools and highly specific and sensitive laboratory tests, constitute the most comprehensive study on the natural evolution of *Trypanosoma brucei gambiense* infection in its human host. At least two alternative natural progressions of HAT to the “classic” fatal one were observed.

## Materials and Methods

### Ethics statement

All samples were collected within the framework of medical surveys and epidemiological surveillance activities supervised by the national HAT control program (NCP). No samples other than those collected for routine screening and diagnostic procedures were collected. All participants were informed about the objective of the study in their own language and signed an informed consent form. This study is part of a larger project aiming at improving HAT diagnosis for which approval was obtained from the WHO (Research Ethics Review Committee) and Institut de Recherche pour le Développement (Comité Consultatif de Déontologie et d'Ethique) ethical committees.

### Study subjects

Within the framework of surveillance activities carried out in February 2004 and May 2009 in the western central part of the Ivory Coast in collaboration with the National Control Program (NCP) and local health structures, the following 50 subjects were re-examined to assess the progression of their HAT status:

- HAT patients diagnosed between 1995 and 1996 in the Sinfra focus who had not been treated after initial diagnosis (*n* = 7)
- HAT patients diagnosed between 2000 and 2007 in the Bonon focus who had not been treated after initial diagnosis (*n* = 4)
- HAT patients diagnosed (18 in first stage, 21 in second stage) between 1995 and 1996 in the Sinfra focus (*n* = 39) who received treatment after initial diagnosis

### Diagnostic tests and clinical examination

Blood (4 ml) was collected in heparinised tubes. A twofold plasma dilution series made in CATT buffer was tested to assess the end titre, i.e. the highest dilution still positive (CATT-P). CATT-P was considered positive if the end titre ≥1/8. CATT is the main serological test used for mass-screening in *T. b. gambiense* endemic areas. All subjects included in the study underwent parasitological examinations by the mini-anion exchange centrifugation technique [15] and by direct microscopical examination of lymph node aspirate when enlarged lymph nodes were present.

As the CATT is known to exhibit false-positive results, Immune trypanolysis tests (TL) were performed on plasma as previously described [16] with LiTat 1.3, 1.5 and 1.6 variable antigen types (VAT) of *T. b. gambiense*. The TL test is highly specific for *T. b. gambiense* and is now routinely used in West Africa in the frame of epidemiological surveillance to better characterise parasitologically unconfirmed CATT-seropositive subjects [17]. Polymerase chain reaction (PCR) using the TBR1/TBR2 primers specific for *Trypanozoon* [18] was performed on DNA extracted from 500 µl of whole blood [19].

For all study subjects, a clinical form was filled out, recording symptoms such as fever, headache, loss of appetite, asthenia, presence of swollen cervical lymph nodes or the following neurological symptoms: daytime somnolence or nocturnal insomnia, presence of the palmomental reflex, sexual activity disturbance, abnormal movements such as tremors and psychiatric disorders such as confusion, agitation, aggressive behaviour or euphoria.

## Results

### Clinical investigations

No neurological disorders specific of the meningoencephalitic stage of the disease were observed in any of the examined subjects. Non-specific clinical signs, such as fever and headache, were frequently reported, in 58% of the treated and 68% of the non-treated study subjects, but the difference was not significant. Enlarged cervical lymph nodes were detected only in one untreated patient from the Bonon focus.

### Serological and parasitological status of treated HAT patients 15 years after diagnosis

In the Sinfra focus, 39 HAT patients diagnosed (CATT on plasma (CATT-P) and parasitologically positive) and treated in 1995–1996 (HAT-treated) were examined in 2009. All had negative results in both parasitological and PCR tests. Results of the CATT-P and trypanolysis test (TL) are given in Table 1. Fourteen (35.9%) patients showed negative results in both CATT and TL tests. Three patients (7.7%) still had positive CATT-P results, while 24 (61.5%) had positive TL results, of which only two were positive for all three variable antigen types (VATs). More stage 2 (P2) HAT-treated patients had positive TL results (17/21, 81%) than stage 1 (P1) HAT-treated patients (7/18, 38.9%), although this difference was not significant (*p* = 0.19, Fisher exact test).

**Table 1:** CATT-P and TL results of the 39 treated HAT cases followed up in 2009 in the Sinfra focus.

Treated HAT P1^1^			Treated HAT P2		
CATT-P^2^	TL^3^	Number	CATT-P	TL	Number
+	+/+/+	1	+	+/−/−	1
+	−/−/−	1	−	+/+/+	1
−	−/−/−	10	−	−/−/−	4
−	+/−/−	3	−	+/−/−	4
−	−/+/−	2	−	−/+/−	6
−	+/+/−	1	−	+/+/−	2
		Total = 18	−	+/−/+	2
			−	−/−/+	1
					Total = 21

1 HAT patients diagnosed and treated in 1995/1996 as first-stage cases.

2 CATT on plasma, considered positive (+) if CATT-P end titres ≥1/8.

3 trypanolysis test, results are given as follows: Litat 1.3/Litat 1.5/Litat 1.6 (+ = positive TL).

### Serological and parasitological status in HAT patients refusing treatment

In the Sinfra focus, seven individuals recorded as subjects 4, 5, 6, 7, 12, 13, and 14 by Jamonneau *et al.*, 2000 [10], still living in the area and never treated for HAT, were re-examined in 2004 and 2009. Parasitological, serological, and PCR results obtained in 1999 [10], 2004, and 2009 are given in Table 2. While trypanosomes were detected in three of these seven patients in 1999, none of them was found to have the parasite by microscopy in 2004 and 2009. While all patients examined in 1999 and 2004 were PCR-positive, they were all PCR-negative in 2009. Three patients had CATT-P positive results in 2009 and six had TL-positive results with two or three VATs. Patient 4 had negative results for all tests in 2009. Patients 5, 6 and 14 became CATT-P-negative but were still TL-positive in 2009. Patients 7, 12 and 13 remained CATT-P-positive and were TL-positive with the three VATs tested in 2009.

**Table 2:** Results of the follow-up of seven untreated patients in the Sinfra focus.

Year	1999^1^			2004				2009			
Patient	CATT-P^2^	T^3^	PCR	CATT-P	TL^5^	T	PCR	CATT-P	TL	T	PCR
4	+	−	+	a^4^	a	a	a	−	−/−/−	−	−
5	+	−	+	+	+/−/+	−	+	−	+/−/+	−	−
6	+	−	+	a	a	a	a	−	+/−/+	−	−
7	+	−	+	+	+/+/+	−	+	+	+/+/+	−	−
12	+	+	+	a	a	a	a	+	+/+/+	−	−
13	+	+	+	+	+/+/+	−	+	+	+/+/+	−	−
14	+	+	+	+	+/−/−	−	+	−	+/+/−	−	−

All patients were positive to the CATT performed on plasma and trypanosomes were detected either in blood or lymph juice when diagnosed between 1995 and 1996.

1 Results from Jamonneau et al. (2000).

2 CATT on plasma, considered positive (+) (i) in presence of a visible agglutination when performed with 5 µl of plasma (1999 and 2004) and (ii) if CATT-P end titres ≥1/8 (2009).

3 Trypanosome in blood and/or lymph fluid (+ = presence, − = absence).

4 absence of the patient.

5 trypanolysis test, results are given as follows: Litat 1.3/Litat 1.5/Litat 1.6 (+ = positive TL).

In the Bonon focus, four untreated HAT patients diagnosed between 2000 and 2007 and still living in the area were re-examined in 2009. Results are shown in Table 3. One patient (BONT4) still had positive microscopy results for both lymph and blood samples tested in 2009. He also had positive results on the CATT-P and TL tests with the three VATs and PCR. The patient continued to refuse to go to the treatment centre where lumbar punctures are performed before initiating treatment. It was therefore not possible to determine the disease stage, although clinical investigations suggest that he was likely still in the first stage. The other three patients diagnosed before 2005 had negative results in both CATT-P and parasitological tests. These three patients were TL-positive with LiTat 1.3 and LiTat 1.6, but negative with LiTat 1.5.

**Table 3:** Results of the follow-up of four untreated patients in the Bonon focus in 2009.

		Results in 2009			
Patient	Diagnosed in	CATT-P^1^	T^2^	TL^3^	PCR
BONT1	2003	−	−	+/−/+	−
BONT2	2000	−	−	+/−/+	−
BONT3	2004	−	−	+/−/+	−
BONT4	2007	+	+	+/+/+	+

All patients were positive to the CATT performed on plasma and trypanosomes were detected either in blood or lymph juice at first diagnosis.

1 CATT on plasma, considered positive (+) if CATT-P end titres ≥1/8.

2 Trypanosome in blood and/or lymph juice (+ = presence, − = absence).

3 trypanolysis test, results are given as follows: Litat 1.3/Litat 1.5/Litat 1.6 (+ = positive TL).

## Discussion

The identification and follow-up over 5–15 years of 11 patients diagnosed with HAT in the Ivory Coast but refusing treatment was a unique opportunity to characterise the diversity of *T. b. gambiense* infection outcomes in its human host. The data presented here – based on clinical, serological, molecular and parasitological investigations, combining field diagnostic tools (mAECT and CATT) and more specific and sensitive laboratory tests (TL and PCR) – challenge the dogma that *T.b. gambiense* infection in humans is 100% fatal.

### Clinical and parasitological cure is associated with a progressive decrease of the serological response

All patients re-examined 15 years after treatment were clinically healthy and parasitologically negative to both mAECT and PCR. Whilst most patients became CATT-P-negative, 61.5% remained TL-positive. This result confirms that *T.b. gambiense*-specific antibodies may remain present in blood for several years after successful treatment [20], [21], [22], [23] and that TL is more sensitive in detecting these antibodies. However, in contrast to what is observed during active disease in which TL reactivity to all three VATs is systematically seen in the Ivory Coast [17], almost all TL-positive treated patients were negative to at least one VAT. Serologically, cure is associated with a decrease of CATT positivity and a progressive loss of reactivity to the different VATs, a process that can last for years.

Since these apparently cured patients had parasitologically negative blood test results, and since there was no clinical suspicion of relapse, for ethical reasons no lumbar puncture was performed to check for the presence of trypanosomes and/or abnormal white cell counts in the cerebrospinal fluid (CSF). We therefore cannot exclude that there were trypanosomes in the CSF, hidden from the peripheral immune system. In this regard, a recent large-scale study carried out in the Democratic Republic of the Congo has shown that in contrast to PCR on blood, PCR on CSF can sometimes remain positive for at least 2 years after apparent successful treatment [24]. These authors concluded that the dogma stating that cure equals parasite elimination may need revision.

### Infection by *T.b. gambiense* is not 100% fatal

Whilst in most patients refusing treatment, infection evolved “classically”, i.e. from stage 1 to stage 2 after 2–4 years [10], eleven patients did not show any appearance of neurological signs. Apart from subject BONT4, diagnosed in 2007 and confirmed to still harbour trypanosomes 2 years later, an apparent parasitological clearance was observed using microscopy after several years in the other ten asymptomatic subjects. Parasitological clearance in these individuals was also suggested by the negative results of the TBR1/2 PCR, although this seemed a longer process. Based on the analysis of the serological response, these subjects becoming apparently aparasitaemic can be divided into two groups.

A first group of seven untreated patients became CATT-P-negative. Six were still reactive with one or two VATs and one was negative to all tested VATs. These individuals displayed the same serological profile as observed in the majority of the cured patients: negative CATT-P results and a progressive loss of reactivity to LiTat 1.3, 1.5 or 1.6 VATs. Thus, clinical, parasitological and serological results strongly argue that self-cure occurred. Scarce and old reports [25], [26], [27], [28] have already described the existence of spontaneous resolution of infections. However, these reports have always been interpreted with caution since at that time microscopic tests were severely impaired by low sensitivity and no serological tests were available [7]. The results presented here, combining both follow-up over 5–15 years and the use of the most sensitive and specific diagnostic tests available, strongly support the fact that spontaneous resolution is a possible scenario of *T.b. gambiense* infection in humans. As for the cohort of cured patients, however, we cannot exclude that latent asymptomatic infections persist in the central nervous system (CNS), since no lumbar puncture was performed in these subjects who were otherwise healthy and negative to all parasitological tests performed on blood. Whereas none of the study subjects reported using traditional medicine, we cannot objectively exclude that they did use plants with potential trypanocidal activity [29].

Three untreated patients remained CATT-P-positive and TL-positive with all three VATs tested. This profile corresponds to the typical serological profile found in HAT patients in the Ivory Coast [17] and to the profile observed in patient BONT4, diagnosed in 2007 and confirmed to still harbour trypanosomes in 2009. These strong long-lasting peripheral serological responses suggest that these persons are asymptomatic carriers who are able to control parasitaemia at levels that are undetectable by microscopy and PCR [30]. Although it is known that antibodies may persist for long periods, it seems unlikely that maintenance of high CATT responses associated with positivity to the three VAT for more than 10 years can occur without some stimulation of the immune system by *T. b. gambiense* antigens. Such individuals are probably not marginal cases as illustrated by the fact that parasitologically non-confirmed seropositive subjects are frequently encountered during medical surveys [17], [31], [32] in different proportions depending on the disease foci [17]. In Bonon for example, trypanosomes were demonstrated in less than 50% of the CATT-P and TL-positive individuals. Likewise, seropositive subjects from the Ivory Coast and Guinea were shown to maintain their serological profile over more than 2 years by longitudinal follow-ups [20], [30]. Because of drug toxicity and costs, most parasitologically unconfirmed seropositive subjects remain untreated. To which extent these individuals may constitute a human reservoir of parasites contributing to the maintenance of transmission in HAT foci is presently unknown and deserves further investigation. It is noteworthy that it was shown that cattle chronically infected with *T.b. brucei* [33] and pigs experimentally infected with *T.b. gambiense* [34], and where trypanosomes are almost undetectable in blood, are still infective for tsetse flies. In this respect, asymptomatic *T.b. gambiense* infection is comparable to the frequent asymptomatic infections occurring with *Trypanosoma cruzi* and *Leishmania* sp., two other human pathogenic members of the *Trypanosomatidae* [35], [36], [37]. A difference however for these parasites, as compared to African trypanosomes, is that they are encountered in their mammalian host as intracellular parasites. Although African trypanosomes are considered to be exclusively extracellular, old and more recent reports exist on putative intracellular amastigote and trypomastigote forms [38], [39]. Whether these forms are viable and/or also exist *in vivo* and whether they may be related to the observed long term seropositivity, remains to be clarified.

### Host and parasite factors underlying HAT clinical diversity remain poorly understood

Altogether, the results presented here strongly suggest that there are at least two possible alternative natural progressions of HAT in addition to the “classic” one (Figure 1): (i) progression to an apparently aparasitaemic and asymptomatic infection associated with strong long-lasting serological responses and (ii) progression to an apparently spontaneous resolution of infection (with negative parasitological and PCR test results) associated with a progressive drop in antibody titres as observed in treated cases. Interestingly, similar courses of infection were also observed when *T.b. gambiense* isolates from the Ivory Coast were used in murine models [40]. This variety in disease outcome may be associated with the genetic variability of the parasite and/or the host [6], [8], [41].

**Figure 1:** “Classic” and possible alternative natural progressions of HAT. Cpl = CATT on plasma, considered positive (Cpl+) if end titres ≥1/8 TL = Trypanolysis test, considered positive (TL+) if positive to at least one variant P = Parasitological investigations in blood and/or lymph fluid (P+ = presence of trypanosome).

Concerning parasite genetic variability, two studies have shown that different *T.b. gambiense* field isolates from the Ivory Coast exhibit contrasting infection patterns in a given mice experimental model and have the capacity to largely influence the host immune response both in terms of quality and quantity [40], [42]. Whether these differences translate directly to humans, however, remains an open question. On the contrary, population genetic studies carried out on trypanosomes from the Ivory Coast and Guinea revealed that *T.b. gambiense* genetic diversity is instead linked with geographic and temporal differentiation processes and did not detect effects on the severity of disease [32], [43], [44]. Trypanosome stocks were repeatedly isolated from several untreated patients included in this study (patients 12, 13, 14, BONT2 and BONT3). Both isoenzyme analysis [45] and microsatellite genotyping [46] have shown that these patients were infected by *T.b. gambiense* group1 that were similar to those from the other HAT patients in the same focus. Whole-genome sequencing is currently underway and will provide an exhaustive genetic characterisation of these strains.

From the host point of view, only very few studies have directly assessed the question of genetic susceptibility in humans, in contrast to the work carried out on inbred strains of mice displaying differences in susceptibility to trypanosome infections [47], [48] and trypanotolerant cattle [49]. It is, however, noteworthy that two studies, one of which was performed in the Sinfra focus in the Ivory Coast and the other in the Democratic Republic of the Congo, have highlighted associations between cytokine gene polymorphisms and a variable risk of developing the disease, thus indicating that the genetic make up of the host may influence infection outcomes [50], [51].

In conclusion, the results presented here, based on the 5- to 15-year follow-up of untreated patients, definitively demonstrate that HAT is not 100% fatal. While this study does not allow a precise evaluation of how frequent self-cure and/or progression to latent asymptomatic infections are, and whether such phenomenon also occur in other HAT foci, a disease course such as these were observed in at least 7 of 53 HAT patients initially refusing treatment in Ivory Coast. Although most of these 53 patients were mainly stage-1 patients suffering from mild symptoms and such infection courses are likely less frequent in stage-2 patients, the fact that sub-clinical and self-resolving asymptomatic infections appear to be long-lasting processes argue in favor of the fact that such individuals may accumulate over time and could thus represent a large fraction of *T.b. gambiense*-infected individuals at a given time in endemic areas. As is widely accepted for rodents and cattle, trypanotolerance also seems of importance in humans. To what extent trypanotolerant persons are involved in the transmission cycle and the respective role of host and parasite factors deserves further investigation.

From our point of view, recognising that trypanotolerance exists in humans is a major step forward for future research in the field of HAT. It has implications both (i) at the intervention level, since these data suggest that latent infections (undetectable by the parasitological tests used in the field) may last for years and thus participate in the maintenance of transmission in endemic areas despite the control measures taken and (ii) at the scientific level, since the trypanotolerant phenotype in humans opens the way to identifying human-specific defence and immune mechanisms involved in the control of *T.b. gambiense* infection and thus new candidate therapeutic or prophylactic targets.
